The article "Methionine-induced regulation of growth, secondary metabolites and oxidative defense system in sunflower (Helianthus annuus L.) plants subjected to water deficit stress" was retracted in 2022. Reasons: compromised peer review; a conflict of interest; concerns about the authorship.

# Methionine-induced regulation of growth, secondary metabolites and oxidative defense system in sunflower (*Helianthus annuus* L.) plants subjected to water deficit stress

**DOI:** 10.1371/journal.pone.0259585

**Published:** 2021-12-09

**Authors:** Gull Mehak, Nudrat Aisha Akram, Muhammad Ashraf, Prashant Kaushik, Mohamed A. El-Sheikh, Parvaiz Ahmad

**Affiliations:** 1 Department of Botany, Government College University, Faisalabad, Pakistan; 2 University of Agriculture Faisalabad, Faisalabad, Pakistan; 3 Instituto de Conservación y Mejora de la Agrodiversidad Valenciana, Universitat Politècnica de València, Valencia, Spain; 4 Botany & Microbiology Department, College of Science, King Saud University, Riyadh, Saudi Arabia; 5 Department of Botany, GDC Pulwama, Srinagar, Jammu and Kashmir, India; Anhui Agricultural University, CHINA

## Abstract

Optimum water availability at different growth stages is one the major prerequisites of best growth and yield production of plants. Exogenous application of plant growth regulators considered effective for normal functioning of plants under water-deficit conditions. A study was conducted to examine the influence of exogenously applied L-methionine on sunflower (*Helianthus annuus* L.) plants grown under water-deficit conditions. Twenty-five-day old seedlings of four sunflower cultivars, FH331, FH572, FH652 and FH623 were exposed to control (100% F.C.) and drought stress (60% F.C.) conditions. After 30-day of drought stress, L-methionine (Met; 20 mg/L) was applied as a foliar spray to control and drought stressed plants. Water deficit stress significantly reduced shoot fresh and dry weights shoot and root lengths, and chlorophyll *a* content in all four cultivars. While a significant increase was observed due to water deficiency in relative membrane permeability (RMP), malondialdehyde (MDA), total soluble proteins (TSP), total soluble sugars (TSS), ascorbic acid (AsA) and activity of peroxidase (POD). Although, exogenously applied Met was effective in decreasing RMP, MDA and H_2_O_2_ contents, it increased the shoot fresh weight, shoot length, chlorophyll *a*, chlorophyll *a/b* ratio, proline contents and the activities of SOD, POD and CAT enzymes in all four cultivars under water deficit stress. No change in AsA and total phenolics was observed due to foliar-applied Met under water stress conditions. Of all sunflower cultivars, cv. FH-572 was the highest and cv. FH-652 the lowest of all four cultivars in shoot fresh and dry weights as well as shoot length under drought stress conditions. Overall, foliar applied L-methionine was effective in improving the drought stress tolerance of sunflower plants that was found to be positively associated with Met induced improved growth attributes and reduced RMP, MDA and H_2_O_2_ contents under water deficit conditions.

## Introduction

Scarcity of water solely and/or in combination with other environmental cues related to soil or atmosphere, decreases rate of growth and yield production of crop plants. Deficiency of water as one of the major limiting factors, adversely affects the life span of plants at different growth stages [1–3]. Different physio-biochemical processes such including water relations, respiration, photosynthesis, stomatal opening, hormonal regulations, protein contents, nutrients status, osmotic adjustment as well as efficiency of photosystems experiences adversaries due to deficiency of water [3–6].

Under water deficit conditions, plants develop mechanisms that could help the plants in survival and improved rate of production [7, 8]. Under deficiency of water, plants upregulate defense mechanism for their survival and get control of increased accumulation of ROS (reactive oxygen species) [8–11]. Owing to drought, the oxidative stress more severely affects the processes taking place in mitochondria and chloroplasts [12, 13]. Due to over-generation of ROS, cell death occurs mainly due to aberration in nucleic acids, DNA, RNA, proteins and vital membranes [14]. Plants can trigger their oxidative defense system to offset stress-induced oxidative stress by increasing the levels/activities of antioxidants [13]. Among enzymatic antioxidants, SOD, POD, POX, CAT and GR are promising ones. However, the non-enzymatic antioxidant compounds include phenolics, tocopherols, glutathione (GSH), AsA and carotenoids [15, 16].

Due to osmotic effect salts dissolved in the soil solution decreases water potential [17]. Moreover, ion specific effect also take place due to high accumulation sodium (Na^+^) and chloride (Cl^-^) ions [18, 19]. Na^+^ inhibits the enzyme activity of many enzymes that require K^+^ for optimal functioning [20–22]. Water stress induces disruption of the K^+^ homeostasis leads to impairment, in root and leaf tissues metabolism. So, tolerant cultivars survive under osmotic stress due to high cytosolic K^+^/Na^+^ ratio in contrast to stress susceptible ones [23, 24].

Due to the unexpected changes in weather and corresponding factors, temperature of the earth is increasing day-by-day, which can cause alarming situation for the production of crops under water deficit conditions. Under such conditions, numerous changes occur in plant metabolism that affect the cell expansion and rate of photosynthesis [25–29]. Moreover, stress-induced change in plasma membrane [30] could be attributable to alteration in the ultrastructure of membrane macromolecules; this leads to poor plant growth and development under water limited regimes [31]. Although water deficiency causes suppression in growth at every stage of a plant, water deficiency particularly at the blossoming stage can cause maximum yield as has already been observed in sunflower plants [32]. At later growth stages, e.g., flowering and seed-ripening, sunflower is much sensitive under water scarce conditions [33]; this causes considerable loss in yield and oil content of sunflower [34, 35]. Thus, practical means need to be implemented to mitigate the adverse effects of drought on sunflower. One of the promising and shot-gun approaches is the exogenous application of different types of organic chemicals both natural and synthetic [36, 37]. Different types of nitrogenous compounds including some promising amino acids are being used these days as growth regulators. Of them, L-methionine has been reported to be an effective regulator of growth and development of plants subjected to environmental cues including drought stress [38]. They observed that in addition to the accumulation of histidine, arginine, proline and threonine, methionine was also increased significantly in drought tolerant sesame [38]. Likewise, previously Kwon, Abe [39] found that overproduction of threonine and methionine established enhancement in saline tolerance of mutant cell line of rice (*Oryza sativa* L.).

Keeping in view the importance of plant growth regulators, it was hypothesized that foliar-applied L-methionine (Met) could improve the growth and metabolism of sunflower plants under stress conditions. Thus, the major objectives of the current study were to evaluate the role of exogenously applied Met in regulating chlorophyll pigments, mechanism of osmoprotection and oxidative defense system of water-stressed sunflower plants.

## Materials and methods

To appraise the interactive effect of water stress and exogenous application of L-methionine on sunflower plants, a pot experiment was carried-out at GC College University Faisalabad, Pakistan with an average atmospheric condition: photoperiod 8.5 h, and RH 70.2%, temperature 35°C. For this purpose, achenes of four cultivars (FH331, FH572, FH652 and FH623) of sunflower were obtained from the Oil-seed Section, Ayub Agricultural Research Institute, Faisalabad, Pakistan. Before sowing, the achenes were soaked in water for 50 min. Plastic pots were taken and each filled with 8000 g sandy loam soil, and 8 achenes were sown in each pot. This experiment was arranged in a completely randomized design with three replicates of each treatment. After 10 days of seed germination, four plants were maintained in each pot after thinning. The pots were covered with an aluminum sheet to protect the plants from rainfall. After 21 days of seed germination, plants were subjected to control (100% field capacity) and drought stress (60% FC). After 30 days of drought stress treatment, L-methionine (20 mg/L) was applied as a foliar spray. A hand plastic sprayer was used for this application. Two plants from each pot were harvested after two weeks of Met application and their fresh and dry weights noted. The remaining plants were used to collect fresh leaf samples and preserved them at -20°C for the determination of the following attributes:

### Chlorophyll contents

Leaf tissue (0.25 g) was ground in 5 ml acetone (80%) and then centrifuged at room temperature. The absorbance of the supernatant was taken at 663 and 645 nm and then chlorophyll *a* and *b* were calculated following Arnon [40].

### Relative water content

Following the protocol developed by Jones and Turner [41], relative water content (RWC) was appraised. From each replicate, a fresh leaf was taken, labeled and weighed for its fresh weight. All the leaves were dipped in de-ionized water for three hours. After this period, turgid weights were noted. All leaf samples were air-dried and shifted into an oven at 70°C for 72 h and then dry weights recorded.

### Relative Membrane Permeability (RMP)

Fresh leaf tissue (0.5 g) was chopped into small pieces and placed them in test tubes each containing 10 ml distilled water. After it, EC_0_ was measured and placed the sample for 24 h at 4°C and determined EC_1_. Then, the samples were autoclaved at 105°C for 20 min and measured EC_2_. Then, RMP was determined using the protocol of Yang, Rhodes [42].

### Proline contents

A protocol established by Bates, Waldren [43] was used to determine free leaf proline contents. For this purpose, 0.5 g fresh leaf was extracted in 3% sulfosalicylic acid. Then, 2 ml of the leaf extract were mixed with ninhydrin (2 ml) and glacial acetic acid (2 ml). Then the samples were heated at 90°C for one hour, ice cooled and added 4 ml toluene to each sample. After it, all samples were vortexed and then their absorbance recorded at 520 nm using a spectrophotometer.

### Glycine betaine (GB) contents

Dried leaf (0.1 g) samples were extracted in distilled water and kept overnight. The sample was centrifuged and 1 ml of 2 N sulphuric acid was added to 1 ml of the filtrate. In a test tube, 0.5 ml of the mixture was taken and reacted with 0.2 ml of potassium tri-iodide. The mixture was shaken, cooled and added 5 ml of 1,2-dichloroethane to it after the addition of 2.8 ml of pre-chilled distilled water. GB contents in the samples were measured following the protocol depicted by Grieve and Grattan [44].

### Malondialdehyde (MDA) contents

Following the method of Carmark and Horst [45], fresh leaf (0.25 g) was extracted with 5 ml trichloroacetic acid (TCA). The mixture was centrifuged at 12,000 x g for 15 min. Then, 1 mL of the supernatant and 4 mL of thiobarbituric acid (TBA) were mixed. The mixture was heated at 95°C for 30 min, later on chilled, and the absorbance was read at 532 and 600 nm using a spectrophotometer.

### Hydrogen peroxide (H_2_O_2_)

Following a procedure proposed by Velikova, Yordanov [46], the samples were prepared using 0.5 g fresh leaf from each treatment. The sample was centrifuged for 15 min at 12,000 x *g*. To 0.5 mL of the supernatant, 1 mL of 1 M potassium iodide and 0.5 mL of potassium phosphate buffer were added, and shaken vigorously. Then, the absorbance of the mixture was read at 390 nm using a spectrophotometer.

### Ascorbic acid (AsA) contents

Ascorbic acid contents were determined following Mukherjee and Choudhri [47]. Leaf sample (0.25 g) was extracted with 6% TCA and then the samples were appropriately centrifuged. Then an aliquot of 2 ml of the filtrate was treated with 1 ml of dinitrophenyl hydrazine. After adding a drop of diluted thiourea to each sample, the mixture was placed in a water bath at 95°C for 15 min. Then, the samples were cooled at room temperature and 5 ml of 9N H_2_SO_4_ were added to each sample. The absorbance of each sample was read at 530 nm using a spectrophotometer.

### Total phenolics

A fresh leaf (0.1 g) was homogenized in 5 ml acetone (80%). After filtration, an aliquot (0.1 ml) was taken in a test tube. Distilled water (2.0 mL) was added to each sample along with 1 ml of the Folin-Ciocalteu’s reagent. Then, 5 ml of 20% sodium carbonate were added to each sample and raised the volume to 10 ml with distilled water. The OD of the mixture was read at 750 nm and total phenolics were calculated following Julkenen-Titto [48].

### Total soluble sugars

A fresh leaf (0.1 g) was placed in a test tube and 3 ml of the anthrone reagent were added to it. Then the mixture was placed on a water bath at 95°C for 15 min and cooled it in a chilled ice bath. Then, the mixture was used to read the absorbance at 625 nm and total soluble sugars determined following Yemm and Willis [49].

### Total soluble proteins

A fresh leaf (0.5 g) was extracted in 5 ml of phosphate buffer (7.8 pH). A reagent was prepared by adding 100 mg Comassie Brilliant Blue G-250 plus, 50 ml (90%) ethanol and 100 ml (85%) phosphoric acid. The mixture was mixed well and filtered three times. This reagent was used for the determination of total soluble proteins following the method of Bradford [50].

### Activities of antioxidant enzymes

The leaf extract prepared for the determination of total soluble proteins was used for the determination of enzymatic antioxidants. A detailed protocol of Chance and Maehly [51] was followed to measure the activity of peroxidase (POD) and catalase (CAT). For POD determination, 0.1 ml of plant extract, 1.0 ml of guaiacol (20 mM), 0.9 ml of H_2_O_2_ (40 mM) and 1.0 ml of phosphate buffer (50 mM) were added, and absorbance read at 470 nm. While for CAT determination, the change in absorbance of the reaction mixture (0.1 ml of enzyme extract + 1 ml of 5.9 mM H_2_O_2_ + 1.9 ml of 50 mM phosphate buffer) was read at 240 nm every 20 s. However, a protocol developed by Giannopolitis and Ries [52] was followed for the determination of the activity of superoxide dismutase (SOD). For this purpose, the enzyme reaction mixture (400 μl distilled water, 250 μl of 50 mM phosphate buffer, 100 μl of 0.1% triton-X, 100 μl of 13 mM L-methionine, 50 μl of 50 μM NBT, 50 μl of 1.3 μM riboflavin and 50 μl enzyme extract) was prepared and noted the absorbance at 560 nm using a spectrophotometer.

### Statistical analysis

A three-way [cultivars (4), drought stress (2) and Met (2)] completely randomized design was employed to determine the analysis of variance of data using Costat V6-303 software. The least significance difference between mean values was calculated at 5% probability level.

## Results

Under drought stress (60% FC), a significant (*P* ≤ 0.001) reduction was recorded in shoot fresh and dry weights of all four cultivars of sunflower (FH331, FH572, FH652 and FH623). Foliar treatment (20 mg/L) of L-methionine (Met) had a significant (*P* ≤ 0.05) influence in improving the shoot fresh weight of all sunflower cultivars. A significant difference was observed among all cultivars in terms of shoot fresh and dry weights. Of all sunflower cultivars, cvs. FH-572 was the highest and FH-652 the lowest in shoot fresh and dry weights under both water stress and exogenously applied Met treatments (Table 1; Fig 1A and 1B).

**Fig 1:** Effect of foliarly treated L-methionine on (A) Shoot fresh weight, (B) shoot dry weights, (C) shoot length and (D) root lengths in sunflower (*Helianthus annuus* L.) plants grown under water deficit condition (Mean ± S.E.).

**Table 1:** Mean squares values (ANOVA) for growth, chlorophyll and oxidative defense system of four cultivars of sunflower (*Helianthus annuus* L.) treated with foliar application of L-methionine (Met) grown under water-deficit stress.

Source of variations	df	Shoot fresh weight	Shoot dry weight	Shoot length	Root length	Chl. a	Chl. b
**Cultivars (Cvs)**	**3**	100.03***	2.777*	129.6***	28.02***	0.074ns	0.005ns
**Drought (D)**	**1**	779.1***	69.26***	6348***	25.88**	2.96***	0.002ns
**Methionine (Met)**	**1**	92.04*	1.077ns	90.75**	4.972ns	0.271**	0.001ns
**Cvs x D**	**3**	78.63**	1.798ns	91.37***	12.98**	0.0009ns	0.011ns
**Cvs x Met**	**3**	14.13ns	0.169ns	12.87ns	2.689ns	0.007ns	0.023ns
**D x Met**	**1**	4.27ns	0.035ns	12ns	3.712ns	0.002ns	0.002ns
**Cvs x D x Met**	**3**	9.65ns	0.215ns	8.125ns	2.631ns	0.072ns	0.008ns
**Error**	**32**	13.19	0.732	9.71	2.441	0.029	0.008
		**Chl. a/b**	**Total Chl.**	**RMP**	**MDA**	**H**_**2**_ **O**_**2**_	**Proline**
**Cultivars (Cvs)**	**3**	0.828ns	0.061ns	103.6ns	18.40***	6456.2**	0.622***
**Drought (D)**	**1**	12.58***	2.784***	4610.1***	13.02*	633.4ns	0.066ns
**Methionine (Met)**	**1**	1.623*	0.238*	609.1**	3.155ns	9092.1**	0.272*
**Cvs x D**	**3**	0.18ns	0.014ns	103.3ns	7.356ns	2214.8ns	0.043ns
**Cvs x Met**	**3**	0.766ns	0.013ns	126.3ns	14.72**	103.9ns	0.338**
**D x Met**	**1**	0.243ns	0.0004ns	32.24ns	40.05***	554.3ns	0.299*
**Cvs x D x Met**	**3**	0.798ns	0.04ns	28.59ns	4.805ns	213.3ns	0.332**
**Error**	**32**	0.315	0.035	76.53	2.612	1074.6	0.053
		**GB**	**AsA**	**Total phenolics**	**TSS**	**TSP**	**SOD**
**Cultivars (Cvs)**	**3**	843.7***	12.76***	82.95**	4508.3***	72.94ns	0.676ns
**Drought (D)**	**1**	96.6ns	8.695**	0.786ns	3345.8*	4226.4**	0.193ns
**Methionine (Met)**	**1**	203.5ns	1.254ns	1.082ns	470.9ns	1989.2*	0.536ns
**Cvs x D**	**3**	158.5*	3.309*	61.08**	1826.7*	1036.6ns	1.633*
**Cvs x Met**	**3**	46.9ns	0.864ns	1.958ns	1400.6*	449.3ns	0.346ns
**D x Met**	**1**	152.4ns	2.868ns	26.86ns	741.4ns	296.7ns	1.366ns
**Cvs x D x Met**	**3**	18.08ns	0.737ns	7.067ns	1491.0*	1545.4*	0.569ns
**Error**	**32**	52.79	0.78	12.48	480.1	468.9	0.543
		**POD**	**CAT**				
**Cultivars (Cvs)**	**3**	0.738ns	0.091**				
**Drought (D)**	**1**	32.06*	0.009ns				
**Methionine (Met)**	**1**	19.91ns	0.003ns				
**Cvs x D**	**3**	8.003ns	0.013ns				
**Cvs x Met**	**3**	2.81ns	0.004ns				
**D x Met**	**1**	2.94ns	0.024ns				
**Cvs x D x Met**	**3**	11.47ns	0.001ns				
**Error**	**32**	7.274	0.015				

**Abbreviations:** Chl, Chlorophyll; RMP, Relative membrane Permeability; MDA, Malondialdehyde; H_2_O_2_, Hydrogen Peroxide; GB, Glycinebetaine; AsA, Ascorbic acid; TSS, Total Soluble Sugars; TSP, Total Soluble Proteins; SOD, Superoxide Dismutase; POD, Peroxidase; CAT, Catalase; ns, No Significant; *, ** and ***, Significant at 0.05, 0.01 and 0.001 levels, respectively.

A significant adverse effect of drought stress was observed on shoot and root lengths of all four sunflower cultivars. Exogenously applied Met was effective in improving the shoot lengths of all four sunflower cultivars under stress and non-stress conditions. The response of all sunflower cultivars varied and cv. FH-572 performed relatively better in terms of shoot length under water-deficit conditions. Of all cultivars, root length of cv. FH-572 was found to be the highest under stress and non-stress conditions (Table 1; Fig 1C and 1D).

Data showed that drought stress (60% field capacity) significantly decreased chlorophyll *a* contents, while chl. *b* remained unaffected in all sunflower cultivars. Application of Met significantly enhanced chl. *a*, and chlorophyll a/b ratio under both stress and non-stress conditions. No significant difference was observed in the four sunflower cultivars in different chlorophyll contents under stress and non-stress conditions (Table 1; Fig 2A–2C).

**Fig 2:** Supplementation of L-methionine restored (A) chlorophyll a, (B) chlorophyll b, and (C) chlorophyll a/b ratio in sunflower (*Helianthus annuus* L.) plants grown under water deficit condition (Mean ± S.E.).

Under water stress, a significant (*P* ≤ 0.001) increase was observed in RMP of all sunflower cultivars. Exogenous application of Met was considerably effective in reducing the RMP under water stress conditions. The response of all sunflower cultivars was almost similar under both stress and non-stress conditions (Table 1; Fig 3A).

**Fig 3:** Foliarly applied L-methionine regulates (A) Relative membrane permeability, (B) MDA content, and (C) H_2_O_2_ content in sunflower (*Helianthus annuus* L.) plants grown under water deficit condition (Mean ± S.E.).

A significant increase in malondialdehyde (MDA) contents, while no change in H_2_O_2_ contents was observed under stress conditions (Table 1; Fig 3B and 3C). Foliar-applied Met was effective in minimizing the MDA and H_2_O_2_ contents particularly in cv. FH623 under both watering regimes. Of all sunflower cultivars, cv. FH572 was the highest in MDA and cv. FH652 in H_2_O_2_ under water stress conditions.

No change in free proline and GB contents was observed in all sunflower cultivars under water stress conditions (Table 1; Fig 4A and 4B). Exogenously applied Met was effective in improving the proline contents in cvs. FH331 and FH623 under control and water stress conditions, respectively. Of all sunflower cultivars, cv. FH652 was the lowest in proline contents. All sunflower cultivars were almost similar in GB accumulation under stress and non-stress conditions.

**Fig 4:** Effect of L-methionine on (A) free proline, (B) GB content, (C) total soluble protein and (D) total soluble sugars in sunflower (*Helianthus annuus* L.) plants grown under water deficit condition (Mean ± S.E.).

A significant increase in total soluble sugars (TSS) and total soluble proteins (TSP) were observed under drought stress conditions in all four sunflower cultivars. However, no significant effect of exogenously applied Met was observed on TSS, while TSP increased significantly (Table 1; Fig 4C and 4D) under both watering regimes. Of all sunflower cultivars, cvs. FH652 and FH623 were better in accumulating TSS, while TSP remained unchanged in all sunflower cultivars.

Ascorbic acid (AsA) contents increased, while no change in total phenolics was observed in the four sunflower cultivars under drought stress conditions. Foliar treatment of Met showed a non-significant effect on AsA and total phenolics of all sunflower cultivars under both watering regimes (Table 1; Fig 5A and 5B). Of all sunflower cultivars, cvs. FH331 and FH623 were relatively better in total phenolics and AsA contents, respectively, under water deficit conditions.

**Fig 5:** External supplementation of L-methionine regulates (A) ascorbic acid and (B) total phenolics in sunflower (*Helianthus annuus* L.) plants grown under water deficit condition (Mean ± S.E.).

The activities of enzymatic antioxidants, (SOD and CAT) were not affected, while the activity of POD increased significantly in all cultivars of sunflower under water deficit conditions. Foliar applied Met had no significant effect on the activities of SOD, POD and CAT enzymes under non-stress conditions, while their activities increased significantly under water deficit conditions due to exogenously applied Met (Table 1; Fig 6A–6C). Of all sunflower cultivars, cv. FH572 was the highest in CAT activity, while no change in the other cultivars for POD and SOD activities was observed under both watering regimes.

**Fig 6:** Effect of foliarly applied L-methionine on activity of antioxidant enzymes (A) SOD, (B) POD and (C) CAT in sunflower (*Helianthus annuus* L.) plants grown under water deficit condition (Mean ± S.E.).

## Discussion

Water is utterly essential for the normal functioning of plant metabolic processes such as photosynthesis, respiration, enzymatic activities, water and nutritional balance, etc. [20]. However, deficiency of water at any stage of plant growth could adversely affect the plant growth and yield production mainly due to dysfunctioning of physiological, biochemical and molecular processes [53–55]. However, the present study was carried-out to assess the effectiveness of exogenously applied L-methionine in upregulation of growth and some key biochemical processes of sunflower (*Helianthus annuus* L.) plants exposed to water-deficit stress. It is now well evident that drought stress can markedly suppress the growth of plants, as already observed in different crops e.g., carrot [56], radish [57], maize [58], sunflower [59], and mung bean [60]. In the present study, drought stress (60% F.C.) significantly reduced the shoot fresh and dry weights of all four cultivars of sunflower (FH331, FH572, FH652 and FH623). However, exogenous application of plant growth regulators is one the effective strategies to minimize stress induced adversaries in plants [61, 62]. Up till now, a number of plant growth regulators, osmoprotectants, mineral nutrients and antioxidants have been applied as foliage application, seed soaking or priming as well as root medium applications on stressed plants [59, 60]. In the present study, foliar-applied L-methionine (Met) at the rate of 20 mg L^-1^ considerably improved the shoot fresh weight as well as shoot length of all four sunflower cultivars. Of all sunflower cultivars, cvs. FH-572 was the highest and FH-652 the lowest in shoot fresh and dry weights under both water stress and exogenously applied Met treatments (Table 1; Fig 1). It is speculated that amino acids can promote growth and safeguard the plants from injuries caused by major abiotic stresses [63]. A prominent role of L-methionine in regulating growth attributes, transpiration, mRNA, protein synthesis and photosynthetic rate has been widely reported [64]. It has been observed that Met has a prominent role in changing the activity of tumor cells (early flowering and heavy branches etc.) leading to better plant growth when histone lysine is converted into Met in plants [65].

High chlorophyll pigments and photosynthetic rate are believed to play major roles in abiotic stress tolerance [25]. Better yield of chlorophyll pigments is usually considered as one of the prospective indicators of drought stress tolerance as observed in a number of studies on different crops e.g., mungbean [66], wheat [67], and chickpea [68]. Water stress is known to cause considerable damages to various physiological and biochemical processes related to photosynthesis, including disruption of stomatal conductance, reduction in chlorophyll content, and interference with photosystem photochemical efficiency and the rate of net assimilation. These can inhibit plant growth resulting in decreased crop production [6, 25, 69]. Met plays an important role in biological events such as methylation and antioxidant properties besides its function in protein synthesis [70]. In the current study, drought stress caused a significant reduction in chlorophyll contents, which may have been due to oxidative stress generated through high accumulation of reactive oxygen species (ROS) as well membrane leakage [11, 25]. Application of Met significantly enhanced chl. *a*, and chl. a/b ratio under both stress and non-stress conditions. However, it is not possible to explain these results as not a single study is available on this aspect in the literature.

Some of the adaptive physiological mechanisms are cell and tissue water conservation which is interlinked with cell membrane stability and endogenous levels of growth regulators [71]. Under water stress, a significant increase was observed in RMP and MDA of all sunflower cultivars. However, exogenous application of Met was considerably effective in reducing the RMP, H_2_O_2_ and MDA contents under water stress conditions. These results clearly suggest that Met application might be involved in maintaining the membrane stability as well as reducing the production of ROS in sunflower plants. Exogenously applied Met was also found to be effective in improving the proline contents in cvs. FH331 and FH623 under control and water stress conditions. It is well evident that osmotic adjustment helps maintain the cell water balance with the active accumulation of solutes in the cytoplasm, thereby minimizing the harmful effects of drought stress [72] and maintaining better growth and yield production as found here in the drought-stressed sunflower plants. In sunflower plants, a significant increase in total soluble sugars (TSS), total soluble proteins (TSP), and ascorbic acid (AsA) were observed under drought stress conditions in all four sunflower cultivars. However, exogenously applied Met accelerated TSP, but a non-significant effect on AsA, total phenolics and TSP was observed under both watering regimes.

Drought stress causes oxidative stress in plants, arising from the excessive production of ROS, which can disrupt the photosynthetic machinery of plants [73]. In the present study, water stress significantly increased RMP and MDA of all sunflower cultivars. However, exogenous application of Met was considerably effective in reducing the RMP, H_2_O_2_ and MDA contents under water stress conditions. The activity of POD increased significantly in all cultivars of sunflower under water deficit conditions. Moreover, foliar-applied Met significantly increased the activities of SOD, POD and CAT enzymes under water deficit conditions. So, high accumulation of antioxidants and sugars might be involved in stress tolerance mechanism of sunflower plants resulting in maintaining better growth and yield production [25, 36].

## Conclusion

In conclusion, drought stress suppressed plant growth and chlorophyll contents, while increased RMP, MDA, TSP, TSS, AsA and the activity of POD enzyme. Overall, exogenously applied Met was effective in minimizing the RMP, MDA and H_2_O_2_ contents, and increasing the plant growth, chlorophyll pigments, proline contents and the activities of SOD, POD and CAT enzymes in all four cultivars of sunflower under water deficit stress. These Met-induced regulations in vital processes were found to be positively associated with better tolerance of sunflower plants to drought stress. So, methionine can be suggested as one of the effective plant growth regulator under stress conditions.

## Supporting information

S1 Data (XLSX)
